# Simulation and Prediction of Fungal Community Evolution Based on RBF Neural Network

This article has been retracted.

**DOI:** 10.1155/2021/7918192

**Published:** 2021-10-08

**Authors:** Xiao-Wei Cai, Ya-Qian Bao, Ming-Feng Hu, Jia-Bao Liu, Jia-Ming Zhu

**Affiliations:** ^1^School of Statistics and Applied Mathematics, Anhui University of Finance and Economics, Bengbu 233030, China; ^2^School of Mathematics and Physics, Anhui Jianzhu University, Hefei 230601, China

## Abstract

Simulation and prediction of the scale change of fungal community. First, using the experimental data of a variety of fungal decomposition activities, a mathematical model of the decomposition rate and the relationship between the bacterial species was established, thereby revealing the internal mechanism of fungal decomposition activity in a complex environment. Second, based on the linear regression method and the principle of biodiversity, a model of fungal decomposition rate was constructed, and it was concluded that the interaction between mycelial elongation and moisture resistance could increase the fungal decomposition rate. Third, the differential equations are used to quantify the competitive relationship between different bacterial species, divide the boundaries of superior and inferior species, and simulate the long-term and short-term evolution trends of the community under the same initial environment. And an empirical analysis is made by taking the sudden change of the atmosphere affecting the evolution of the colony as an example. Finally, starting from summer, combining soil temperature, humidity, and fungal species data in five different environments such as arid and semiarid, a three-dimensional model and RBF neural network are introduced to predict community evolution. The study concluded that under given conditions, different strains are in short-term competition, and in the long-term, mutually beneficial symbiosis. Biodiversity is important for the biological regulation of nature.

## 1. Introduction

The carbon cycle is an important part of life on earth, where the decomposition of compounds allows carbon to be renewed and used in other forms [1]. The key component of this process is the decomposition of plant materials and wood fibers. Related studies have found that the decomposition rate of fungi, a key factor in the decomposition of plant materials and wood fibers, is influenced by temperature, humidity, time, growth rate, mycelial density, and moisture tolerance [2, 3]. And slow-growing fungi are more likely to survive and grow in the environment of humidity and temperature changes, while faster-growing fungi are less resistant to the same environmental changes [4]. At the same time, the decomposition rate of fungi determines the biomass and nutrient content of the forest surface and significantly affects the physical and chemical properties of the soil. By exploring the mycelial elongation rate of fungi and the moisture resistance of fungus, it is possible to reveal the important role of fungi's decomposition mechanism of plant material and wood fiber, as well as the mutual adaptation of coupling modes between different species combinations in biodiversity [5].

He selected the suitable tree species of karst natural community habitat, Constructus and Yungui gooseberry as the research object to investigate how AM fungi regulate soil litter to achieve nutrient release and change soil properties under competitive conditions [6]. Zhang investigated the correlation between the culture products of corn stover in four treatments, basic properties, material content and biological enzyme activities, and the dynamic change pattern of the humus-like composition of culture products [7]. To investigate the effect of endophytic fungi on the decomposition of apoplasts, Chen investigated the effect of endophytic fungi on the decomposition of apoplasts by using different sampling methods and selecting endophytic fungi with different dominance to participate in different community construction [8]. By combining indoor culture experiments and field experiments, Tan investigated the changes of soil microbial biomass, enzyme activities related to soil organic carbon decomposition, and the effects of ectomycorrhizal fungi community structure and diversity, and then analyzed the role of ectomycorrhizal fungi in forest soil organic carbon decomposition [9].

Under natural conditions, microorganisms do not degrade apoplankton independently, but the interactions between decomposer groups and their components cannot be ignored, but due to the complexity of the interactions between microorganisms, soil and apoplankton quality, this aspect has not been well studied. Most of the studies on fungal decomposition and community evolution are based on the biological level and are not well integrated with mathematical models. The data in this paper are from real experimental data, which are reliable and can be closer to the complex natural conditions.

In this paper, first, a mathematical model of the relationship between the decomposition rate of fungal species and fungal species was established based on the experimental data of decomposition activities of various fungi. Second, based on the principle of biodiversity, a linear regression method is used to construct a model of fungal decomposition. Then, using differential equations, a dynamic model of fungal competitiveness was established and empirically analyzed. Finally, the three-dimensional model and RBF neuron network were combined to predict the evolution of the community.

## 2. Basic Assumptions

The research question comes from Question A of the 2021 American College Students Mathematical Modeling Competition, and the data comes from National Center for Biotechnology Information. To explore the above issues, we make the following assumptions: (i) it is assumed that the substances produced by fungal decomposition have no significant impact on itself and the surrounding environment. (ii) It is assumed that only fungi participate in the decomposition process, and other microorganisms do not participate in the decomposition of the compound. (iii) The decomposition of plant material and wood fiber is independent of each other. (iv) It is assumed that the main factors affecting the shape of the fungus that affect the decomposition rate are the fungal hyphae elongation and moisture resistance, and the influence of other factors is negligible. (v) In the competition of fungi, the influence of fungal aerobic respiration, anaerobic respiration, or anaerobic respiration on the decomposition rate is not considered.

## 3. Construction of Fungal Decomposition Model Based on Multiple Linear Regression Method

### 3.1. Research Ideas

To describe the decomposition of organic matter by a variety of fungi, this paper selects seven common fungi as the research object, takes Chinese fir as an example to be decomposed, and constructs a fungal decomposition model [10–12]. By consulting the relevant information, we found that temperature, humidity, colony abundance, time, soil sulfur and phosphorus content, mycelial elongation, and moisture resistance are the main factors affecting the decomposition rate of fungi, so we set them as independent variables and use *K*, *H*, *N*, *T*, *P*, *G*, and *R* to represent, respectively. Besides, we set the mass loss rate of each patch of plant per unit time as the dependent variable, denoted by V. The method of multiple linear regression is used to study the decomposition activity of fungi.

### 3.2. Analysis Steps

#### 3.2.1. Construct a Multiple Linear Regression Model

In this paper, 7 strains of AM fungus, Cladosporium, Trichoderma, Aspergillus flavus, Alternaria spp, Penicillium, and Chaetomium vulgaris were mixed [13], and they were simultaneously inoculated on a petri dish with Chinese fir as the decomposed substance. The experimental data was collected in one week and lasted for 12 weeks. Under the conditions of controlling the temperature and humidity of each group of experiments, the fungus' decomposition activity on the substrate was studied [14].

Standardize the data obtained in the experiment to eliminate the influence of dimensions on the model and use the data to construct a multiple linear regression model.

(1) $$\begin{array}{c} V=a+bK+cH+dT+eS+fG+gR. \end{array}$$

Since this article is seven sets of parallel experiments under the control of temperature *K*, humidity *H*, and fungal richness *N*, the multiple linear regression models of each group can be obtained:

(2) $$\begin{array}{c} \left\{\begin{array}{c} V_{1}=-1.062-0.056K+1.093H-0.212T+0.218P-0.0416G-1.041R,N=1,\\ V_{2}=-1.173-1.041K-1.043H-0.031T+0.237P+2.153G-1.092R,N=2,\\ V_{3}=-0.159+0.483K-1.224H-0.435T-0.083P-1.228G-1.059R,N=3,\\ V_{4}=0.338+2.087K-1.006H-0.052T-0.163P+2.221G+0.162R,N=4,\\ V_{5}=1.387+1.607K-1.020H+0.690T+0.286P+1.156G-1.241R,N=5,\\ V_{6}=1.710+1.609K-0.183H-0.039T+0.189P+0.376G-0.197R,N=6,\\ V_{7}=0.450-0.231K+0.144H-0.058T+0.1429P-0.107G-0.317R,N=7. \end{array}\right. \end{array}$$

To obtain a fungal decomposition rate model closer to the natural environment, this paper uses the entropy method to weight the above equations to eliminate the influence of colony richness *N* on the difference in fungal decomposition rates between the experimental groups to meet the needs of biodiversity.

#### 3.2.2. Entropy Method

By calculating the information entropy of each indicator in the indicator system and determining the weight of the indicator according to the relative change degree of the indicator and the contribution rate to the overall system, it is a method of combining static weighting and dynamic weighting. If the information entropy is smaller, the disorder degree of the information is lower, the utility value of the information is larger, and the weight of the index is larger. Specific steps are as follows:

(3) $$\begin{array}{c} X={\left(x_{ij}\right)}_{mn},\text{namely},X=\left(\begin{array}{ccc} x_{11} & \cdots & x_{1n}\\ \vdots & \ddots & \vdots \\ x_{m1} & \cdots & x_{mn} \end{array}\right). \end{array}$$

(4) $$\begin{array}{c} P\left(x_{ij}\right)=\frac{x_{ij}^{\prime }}{\sum \begin{array}{c} m\\ i=1 \end{array}x_{ij}^{\prime }}. \end{array}$$

(5) $$\begin{array}{c} h_{j}=-k\sum \begin{array}{c} n\\ i=1 \end{array}P\left(x_{ij}\right)\ln P\left(x_{ij}\right),j=1,2,\cdots ,n. \end{array}$$

**Step 1 .**

Define the initial evaluation matrix.

**Step 2 .**

Calculate the ratio of the index value *P*(*x*_*ij*_).

**Step 3 .**

Calculate the entropy value of each index.

Among them, *P*(*x*_*ij*_) represents the corresponding value, *K* > 0, generally take *K* = 1/ln*k*, so 0 ≤ h_*j*_ ≤ 1. The greater the degree of difference between the evaluation, indicators *x*_*ij*_ the greater the contribution rate of the indicator to the entire indicator system and the greater the weight assigned.

(6) $$\begin{array}{c} \omega_{j}=\frac{h_{j}}{\sum \begin{array}{c} n\\ j=1 \end{array}h_{j}},j=1,2,\cdots ,n. \end{array}$$

**Step 4 .**

Calculation of index weight.

The weight of the indicator reflects the degree of influence of the evaluation indicator on the overall performance.

To sum up, when *N* = 1, 2, 3, 4, 5, 6, 7 the weight assigned to each group should be (1.424, 1.729, 1.865, 1.870, 1.885, 1.918, 1.930).

That is, the relationship between the overall fungal decomposition rate and the fungal decomposition rate between groups is

(7) $$\begin{array}{c} 1.424V_{1}+1.729V_{2}+1.865V_{3}+1.870V_{4}+1.885V_{5}+1.918V_{6}+1.930V_{7}. \end{array}$$

Substituting the equations of the above experiment to obtain the decomposition rate model of fungi on fir in the presence of multiple fungi is

(8) $$\begin{array}{c} V=-1.703+2.081K-1.334H-0.046T+0.356P+2.128G-1.093R. \end{array}$$

### 3.3. Conclusion Analysis

It can be found from equation (12) that when the colony abundance *N* = 7, it has a greater impact on the overall fungal decomposition rate, and when *N* = 1, it has a small impact on the overall fungal decomposition rate. To better adapt to the biodiversity of nature, expand the number of studies on colonies, and further explore the impact of biodiversity on fungal decomposition activities, this paper sets a dummy variable *D*_1_. The colony with *N* > 2 is defined as a multicolony group and *D*_1_ = 1 is assigned; the colony with *N* = 1, 2 is defined as a single colony, and the value is *D*_1_ = 0.

(9) $$\begin{array}{c} D_{1}=\left\{\begin{array}{cc} 0 & N=1,2,\\ 1 & N>2. \end{array}\right. \end{array}$$

The average value of the fungal decomposition rate in each group of experiments is selected to indicate the size of the fungal decomposition rate under different colony richness when the temperature, humidity, and other variables are unchanged. Introduce dummy variables in the form of addition, and establish a unary linear model of fungal decomposition rate and colony richness:

(10) $$\begin{array}{c} V=a+bN+D_{1}. \end{array}$$

Substituting the standardized decomposition rate data into equation (10), the equation of decomposition rate and colony richness is obtained as:

(11) $$\begin{array}{c} V=4.9671+0.3452N+1.0387D_{1}. \end{array}$$

The regression results show that the decomposition rate is positively correlated with the colony abundance, and the coefficient before the dummy variable *D*1 is positive, indicating that the multicolony community is beneficial to the decomposition of fungi, that is, the decomposition rate will be significantly increased under the condition of multiple colonies.

From equation (13), it can be found that the fungal decomposition rate is related to temperature, humidity, decomposition time, soil antibiotic content, mycelial elongation, and moisture resistance.

In summary, in a variety of bacterial communities, the decomposition rate of fungi will be significantly increased. Therefore, under the conditions of coexistence of multiple fungi, higher temperature, higher soil phosphorus and sulfur content, and faster growth rate of fungi, the decomposition rate of fungi increases; in the presence of single fungi, higher humidity, longer decomposition time, and higher humidity resistance under the conditions, the decomposition rate of fungi slows down [15–18].

## 4. Construction of a Decomposition Rate Model Based on the Interaction between Fungi

### 4.1. Research Ideas

The rate of change of temperature and humidity has a certain relationship with the vitality of fungi [19]. According to Lustenhouwer et al., the relationship between mycelial elongation and wood decomposition rate is approximately positive and linear; under logarithmic transformation, the relationship between moisture tolerance of different fungi and the final wood decomposition rate is also approximately positive and linear. It can be inferred that there may also be a linear relationship between the moisture resistance of different fungi and the elongation of their hyphae.

Therefore, this paper will use the characteristics of hyphae, elongation, and moisture resistance of different types of fungi to combine the types of fungi. First, we establish a univariate linear regression model to study the relationship between the moisture tolerance of different fungi and the hyphae elongation; second, the two characteristics of fungi are combined under the condition of keeping the fungal decomposition rate constant, that is, the hyphae extension rate represents moisture resistance; finally, substituting the unary linear model into the above fungal decomposition rate model to obtain a modified model—a decomposition rate model based on the interaction between fungi.

### 4.2. Analysis Steps

Under the condition that the decomposition rate of fungi remains unchanged, the relevant data of mycelial elongation and moisture resistance are obtained through web crawling and standardized processing, and a unary linear regression model of mycelial elongation and moisture resistance is constructed:

(12) $$\begin{array}{c} R=a+bG. \end{array}$$

Using SPSS25 software to fit the equations of mycelial elongation and moisture resistance, as shown in Figure 1.

(13) $$\begin{array}{c} R=-0.981G+1.45. \end{array}$$

Thanks for the suggestion, this sentence is revised to: Substitute the above results into the fungal decomposition rate model in section 3.3.2, and get an improved model based on the different interactions among hyphae, elongation, and moisture resistance:

(14) $$\begin{array}{c} V=-1.231+2.018K-0.533H-0.346T+1.056P+1.119G. \end{array}$$

### 4.3. Conclusion Analysis

The change of environmental temperature and humidity is related to the vitality of fungi, that is, it will affect the growth rate of fungi. The decomposition rate of fungi is positively correlated with the growth rate and negatively correlated with the humidity resistance. Under the condition of controlling the decomposition rate unchanged, the fungus growth rate and humidity resistance are combined. It was found that there was a significant negative correlation between the growth rate and moisture tolerance of the fungus, and the interaction between the growth rate and moisture tolerance of the fungus had a positive effect on its decomposition rate.

## 5. Construction of Competitive Dynamic Model Based on Differential Equations

### 5.1. Research Ideas

Different fungi have different moisture resistance, so their mycelial elongation rate or growth rate is different in the same environment [20]. When the size of each colony is different, the limited survival resources will not get a reasonable and even distribution, and the competition relationship between the populations will occur, that is, the interaction [21–25]. The dynamic model is a model that describes the characteristics of the system related to time changes and the environment of the event. It can explore the overall behavior of the system, reduce the complexity of the system with the help of state diagrams or sequence diagrams, and can be completed while monitoring whether the conceptual system has defects. And show the internal operating mechanism of the system in detail [26].

Based on the above analysis, this paper firstly quantifies the internal interaction, namely, establishes a competitive dynamic model to simulate the long-term and short-term evolution trends of the community under the same initial environment under the premise of dividing the boundary between the advantages and disadvantages of the bacteria [27]. Second, consider the sudden external atmospheric changes. The overall impact is to explore the susceptibility of colony evolution to rapid environmental fluctuations.

### 5.2. Analysis Steps

#### 5.2.1. Comparative Analysis

According to the data of changes in the mycelial elongation of each fungus under different temperature and humidity conditions, a scatter plot was drawn with the mycelial elongation as the dependent variable, and temperature and humidity independent.

Variables are shown in Figures 2 and 3.

It can be seen from the above figure that the influence trends of temperature and humidity on different strains are roughly similar, but there are still some differences. To observe the degree of difference more intuitively, this paper selected two fungi from the aspects of temperature and humidity for comparison, to amplify the similarities and differences of the impact of environmental changes on different fungi, as shown in Figures 4–9.

It can be seen from the comparative analysis graph that the overall trend of the sensitivity of different fungi to changes in the external environment is relatively consistent, and all of them can fit the cubic linear equation with a higher coefficient of determination. The impact of the environment on different strains is more significant, that is, under the same external environment, different fungi have different hyphae elongation rates, which in turn creates a competitive relationship between colonies.

#### 5.2.2. Model Construction under General Conditions

The density of the hypha is equal to the ratio of the length of the hypha to the quality of the soil, which describes the density of fungal growth horizontally and can represent the growth scale of the colony. This article is represented by *W*.

According to the above temperature and humidity curve, the evaluation model is introduced to evaluate and score the competitiveness of different fungi, and the competitiveness ranking of each strain is obtained, as shown in Table 1.

According to the size of the competitive ranking, the bacteria are divided into two categories, A and B, based on the value equal to 0.5.

Type A fungi: the competitive ranking is less than 0.5, and it is greatly affected by temperature and humidity. It has greater hyphae elongation and hyphae density at the optimum temperature. This article defines it as an inferior strain.

Type B fungi: competitive ranking is greater than or equal to 0.5 and is less affected by temperature and humidity. It has low hyphae elongation and hypha density at the optimum temperature. This article defines it as a dominant species.

To explore the dynamic changes of the mycelial density D of these two types of bacteria under the long-term and short-term trends under this competitive situation, this paper uses *A*(*t*) and *J*(*t*) to indicate the density of hyphae of type A species and type B species, setting the initial temperature of the fungus to 22°C and 55% humidity under general conditions in week *t*.

- In the long-term process, from the time span of the 1st to 12th week, the following differential equations are obtained using experimental data:

(15) $$\begin{array}{c} \left\{\begin{array}{c} \frac{dA\left(t\right)}{dt}=-aJ\left(t\right),\\ \frac{dA\left(t\right)}{dt}=-bA\left(t\right),\\ A\left(0\right)=0.2475,J\left(0\right)=0.5570. \end{array}\right. \end{array}$$

(16) $$\begin{array}{c} A\left(t\right)-A\left(0\right)=-a\sum \begin{array}{c} t\\ n=1 \end{array}J\left(n\right). \end{array}$$

(17) $$\begin{array}{c} J\left(t\right)-J\left(0\right)=-b\sum \begin{array}{c} t\\ n=1 \end{array}A\left(n\right). \end{array}$$

At week 12:

(18) $$\begin{array}{c} A\left(t\right)=0.2063,J\left(t\right)=0.7640. \end{array}$$

(19) $$\begin{array}{c} \overset{t}{\underset{n=1}{\sum }}A\left(n\right)=0.2269\times 12=2.4958. \end{array}$$

Substituting the above formula into equation (17), we can get

(20) $$\begin{array}{c} -2.4958b=0.7640-0.5557,\text{namely},\;b=0.0835. \end{array}$$

Because *b* < 0, there is a coexistence relationship between A and B species in the long run.

(ii) In the short-term process, from the time span of the 1st to 5th week, the following differential equations are obtained using experimental data

(21) $$\begin{array}{c} \left\{\begin{array}{c} \frac{dA\left(t\right)}{dt}=-aJ\left(t\right),\\ \frac{dA\left(t\right)}{dt}=-bA\left(t\right),\\ A\left(0\right)=0.2475,J\left(0\right)=0.5570. \end{array}\right. \end{array}$$

(22) $$\begin{array}{c} A\left(t\right)-A\left(0\right)=-a\overset{t}{\underset{n=1}{\sum }}J\left(n\right)=-0.2475. \end{array}$$

(23) $$\begin{array}{c} J\left(t\right)-J\left(0\right)=-\text{b}\overset{t}{\underset{n=1}{\sum }}A\left(n\right)=-0.5570. \end{array}$$

At week 5:

(24) $$\begin{array}{c} A\left(t\right)=0.1633,J\left(t\right)=0.4783. \end{array}$$

(25) $$\begin{array}{c} \overset{t}{\underset{n=1}{\sum }}A\left(n\right)=0.2054\times 5=1.027. \end{array}$$

Substituting the above formula into equation (23), we can get

(26) $$\begin{array}{c} -1.027b=0.4783-0.5570,\text{namely},\;b=0.0766. \end{array}$$

Because *b* > 0, there is a competitive relationship between A and B strains in the short term.

In summary, under the conditions of a temperature of 22°C and a humidity of 55%, the A strain and the B strain have short-term competition and long-term coexistence.

#### 5.2.3. Model Construction under Burst Conditions

In the absence of human interference, the changes in the external environment are usually relatively stable, but there will also be certain emergencies [28–30], in which atmospheric changes dominate. Therefore, the following will study the overall impact of atmospheric changes on the interaction between different species of fungi, select temperature and humidity as the main factors affecting the atmospheric level, and still use the mycelial density to represent the growth scale of the colony.

First of all, based on the example of B-type strains, which are dominant strains, a binary linear regression equation with hypha density as the dependent variable and temperature and humidity as independent variables is established using standardized related data.

It can be seen from Table 2 that the model determination coefficient *R*_2_ is 0.087, indicating that the degree of fit is very small, and the *P* values of the coefficients are all greater than 0.05, indicating that the effect of independent variables in the model is not significant. Therefore, the binary linear regression equation is not suitable to explain this problem. This article will consider building a fitting model in a three-dimensional space.

Combine the temperature and humidity data to determine the plane corresponding to each value of the mycelium density, use Matlab software to build a three-dimensional fitting model, as shown in Figure 10.

From Table 3, it is clear that the SSE value of the dynamic model based on the dominant species is extremely small and negligible, and the correlation coefficient *R*-square value is 1, indicating that the model fits well and is able to explain and portray the overall effect of fungal atmospheric changes on the interaction between dominant fungi.

Similarly, the three-dimensional fitting model of atmospheric changes on the class A strain, i.e., the inferior strain, can be obtained, and the results are shown in Figure 11.

Thus, as shown in Table 4, the SSE numerical disadvantage dynamic model-based species can be ignored, the correlation coefficient *R*-square value of 1 indicates that the model fits well the effect, and can be interpreted to characterize changes in the atmosphere between disadvantage fungal fungi are mutually effect.

In summary, by constructing a dynamic model of the influence of temperature and humidity on mycelial density in a three-dimensional space, it is possible to reveal the natural law of interaction between atmospheric changes on different types of fungi and to explore the overall trend of atmospheric changes on the evolution of colonies.

### 5.3. Conclusion Analysis

Changes in the atmospheric environment mainly lead to changes in external temperature and humidity, which in turn affect the initial mycelial density *D* of the superior and inferior strains. Under the disturbance of rapid environmental fluctuations, it is possible that the original dominant strains will gradually weaken or even become inferior strains [31]. The conclusions on the sensitivity of colony evolution to rapid environmental fluctuations are specifically analyzed in this paper in conjunction with the models in Sections 5.2.2 and 5.2.3.

When the initial ambient temperature is 22.5°C and the humidity is 55%, the verification of the competitive dynamic model is constructed in Section 5.2.2. It is known that the relationship between A and B species is a state of short-term competition and long-term mutually beneficial symbiosis, and in the end, B species becomes the dominant species.

When the external environment changes, i.e., the temperature and humidity of the living environment of A and B bacteria change, according to the three-dimensional model constructed in Section 5.2.3, their respective mycelial density *D* will also change in the initial situation.

When the temperature changed to 16.6°C and the humidity changed to 32%, the initial mycelial densities corresponding to the A and B strains were 0.38 and 0.27. We applied the competitive dynamics model to simulate the evolution of the community and obtained that the mycelial densities corresponding to the moment of equilibrium point for A and B fungi were 0.47 and 0.26, respectively. In this case, the class A fungi became the dominant species, in contrast to the original environmental conditions in which they were the weaker species.

Based on the above conclusions, it can be concluded that changes in the environment have a greater impact on the interrelationship between strains, and one manifestation of which is that they change the status of dominant and inferior strains. But in the overall situation, their interrelationship is all about short-term competition and long-term mutually beneficial symbiosis [32].

## 6. Prediction of Relative Advantages and Disadvantages among Species

### 6.1. Research Ideas

Due to the rich biodiversity in nature, the advantages and disadvantages of each species or combination of species are always relative [33–35]. From the abovementioned community evolution, with the change of time, the dominant species may become the inferior species, and predicting the relative advantages and disadvantages among species can determine the dominant species, which is conducive to exploring the inner mechanism of nature's superiority and inferiority.

### 6.2. Prediction of Relative Strengths and Weaknesses

By reading various references [36–41], soil temperature, humidity, fungal species, and initial temperature and humidity of five different environmental types with a representative starting point in summer were collected in this paper [42], as shown in Table 5. Where *x*_1_, *x*_2_, *x*_3_, *x*_4_, *x*_5_, and *x*_6_ denote temperature (°C), humidity, fungal species, initial temperature and humidity duration (weeks), equilibrium temperature (°C), and equilibrium humidity, respectively.

From the three-dimensional model of mycelial density and temperature and humidity in Section 5.2.3, it is known that if any combination of temperature and humidity is given, class A and class B strains will have corresponding initial mycelial densities, respectively, and our summary data is shown in Table 6. Where *x*_7_, *x*_8_, *x*_9_, and *x*_10_ denote initial mycelial density of class, A fungi initial mycelial density of class, B fungi mycelial density of class A fungi, in equilibrium and mycelial density of class B fungi in equilibrium, respectively.

From the data in the table, it can be seen that when the temperature is suitable and the humidity is lower, the mycelial density of the A strain is greater than that of the B strain, and the growth rate is faster. At this time, it is the dominant strain. When the temperature is suitable and the humidity is higher, the mycelial density of the B strain is higher than that of the A strain, and the growth rate is faster. At this time, it is the dominant strain.

On the whole, the B strains are less affected by the environment, the mycelial elongation rate is more stable, and the relative advantage is higher. However, due to the continuous changes of the environment over time, the B strain may evolve into a weak strain under special environmental conditions. On the contrary, the A inferior strain may also become a dominant strain.

If there are only a few species of bacteria in the soil, the growth and reproduction of fungi will be greatly affected by environmental changes, and the abundance of colonies will also be affected to a certain extent. If many strains of fungi are present in the soil, the environment, fungi, and fungus are predicted to establish a relationship between their strengths and weaknesses in the colony. In other words, when the environment changes, each species of fungus can complement each other in dynamics and ensure the biodiversity in the soil. After a period of time, the overall size of the colonies of various fungi and the abundance of the colony in the soil remained relatively stable, that is, in the evolution of the community, the various bacterial species compete in the short term, while the long-term different bacterial species present mutually beneficial symbiosis This situation reflects the diversity and richness of biodiversity.

## 7. Biodiversity Prediction Based on RBF Neuron Networks

### 7.1. Research Ideas

It can be seen from the above that the rapid fluctuation of the external environment will affect the vitality of fungi. At the same time, the interaction between different bacterial species will also affect the colony size of each bacterial species.

### 7.2. Analysis Steps

From the above, it can be seen that the status of superior and inferior strains may be interchanged when the environment is changed, and at this time, the abundance of colonies will be affected to some extent. Diverse fungal communities are more “disturbance resistant” and “resilient” when considering the possibility of varying degrees of variability in the local environment, i.e., differences in initial conditions. That is, if the diversity of the fungal community is lost, the ecosystem can still be restored under certain natural laws.

Construction of neuronal network models. The multiple linear regression model has strong correlation between variables, i.e., high multicollinearity, so the accuracy of the model is still lacking. Considering this effect, we use RBF neural network algorithm to implement the prediction model with the help of Matlab software to achieve better prediction results [43].

RBF neural network has strong approximation ability, classification ability, and learning speed. Its working principle is to regard the network as an approximation to an unknown function. Any function can be expressed as a weighted sum of a set of basis functions, that is, the transfer function of each hidden layer neuron is selected to form a set of basis functions to approximate the unknown. Build a neural network model and function. The RBF artificial neural network consists of an input layer, a hidden layer, and an output layer.

Build a general model: set the input layer as *X* = [*x*_1_, *x*_2_, ⋯, *x*_*n*_], and the actual output layer as *Y* = [*y*_1_, *y*_2_, ⋯, *y*_*p*_]. The input layer realizes the nonlinear mapping from *X* to *R*_*i*_(*X*), the output layer realizes the linear mapping from *R*_*i*_(*X*) to *y*_*k*_, and the output of the *k*-th neuron network in the output layer is

(27) $$\begin{array}{c} {\hat{y}}_{k}=\overset{m}{\underset{i=1}{\sum }}w_{ik}R_{i}\left(X\right),k=1,\cdots ,p. \end{array}$$

In equation (27), *n* is the number of input nodes, and *m* is the number of hidden layer nodes; *p* is the number of output layer nodes; *w*_*ik*_ is the connection weight between the *i*-th neuron in the hidden layer and the *k*-th neuron in the input layer; *R*_*i*_(*X*) is the hidden layer the action function of the *i*-th neuron in the layer, namely,

(28) $$\begin{array}{c} R_{i}\left(X\right)=\exp\left(-{\left\|X-C_{i}\right\|}^{2}/2\alpha_{i}^{2}\right),i=1,\cdots ,m. \end{array}$$

In equation (28), *X* is the *n*-dimensional input vector; *C*_*i*_ is the center of the *i*-th basis function, a vector with the same dimension as *X*; *α*_*i*_ is the width of the *i*-th basis function; *m* is the number of perceptual units (the number of hidden layer nodes); the norm of the vector ‖*X* − *C*_*i*_‖, which usually represents the distance between *X* and *C*_*i*_; the unique maximum value of *R*_*i*_(*X*) at *C*_*i*_. As ‖*X* − *C*_*i*_‖ increases, *R*_*i*_(*X*) decays rapidly to 0.

For a given input, only a small portion near the center of *X* is activated. Once the clustering centers *C*_*i*_, weights *w*_*ik*_, and *α*_*i*_ of the RBF network are all determined, the corresponding output values of the network can be given for a certain input.

In this paper, there are 6 independent variables and 1 dependent variable, the number of input neurons is taken as 6, the number of output neurons is taken as 1, and the number of neurons in the middle hidden layer is 0. The RBF network will be taken adaptively during the training process.

Use the data in Table 7 to fit the RBF neural network model to predict the decomposition effect of biologically diverse colonies when the local environment has different degrees of variability.

The data were imported into Matlab, and RBF neural networks were performed to fit and combine the predictions. The predictions were compared to single strain conditions to give an arbitrary combination of six initial factor values for colonies with species diversity.

For example, growth rate: 6.16; mycelial density: 0.04; humidity tolerance: 1.52; sulfur and phosphorus content: 46.6; temperature: 23.55; humidity: 0.91, enter code: *p*_*i*_ = [6.16 0.04 1.52 46.6 23.55 0.91].

The predicted value of decomposition rate *t* is 0.31, which is higher and better than the decomposition rate in the case of a single strain.

### 7.3. Conclusion Analysis

Based on the results of the above runs, we can find that the higher the species richness, the higher the decomposition rate. Because different species have different factors such as its mycelial growth rate and growth rate under different environmental conditions, i.e., different rates of decomposition of dead branches and leaves [44]. When the ambient temperature changes abruptly, the A class strains are affected more by weak strains, while the B class strains are affected less as the dominant strains, with a diversity of strains can complement each other between the AB class strains, the overall decomposition rate will not appear too big fluctuations, even if the community is affected more, it can gradually recover to the original level with time. Whereas a single strain is more affected by environmental changes, no complementary strain compensates for the decreased part of the decomposition rate [45]. In addition when it is affected more, it is less resilient than colonies with material diversity. It is thus clear that biodiversity is important for the automatic balance of biological regulation in nature.

## 8. Conclusion

After our reasonable and rigorous model analysis, it was concluded that the decomposition rate of fungi was affected by temperature, humidity, colony abundance, time, soil sulfur and phosphorus content, mycelial elongation rate, and moisture tolerance. Under the given temperature and humidity conditions, different fungi have different mycelial densities, while they show competitive relationships in the short term and mutually beneficial symbiotic relationships in the long term. Different fungi are sensitive to environmental changes, so when environmental conditions change, the original dominant species may become the inferior species. For colonies with high species richness, there are dominant and inferior species in the colony, regardless of environmental changes. They have complementary strengths and weaknesses, and the rate of decomposition is dynamically balanced over time by the combined action of multiple fungi. In addition, plant communities are highly resistant to disturbance and recovery, so biodiversity provides stability to ecosystems.

## Figures and Tables

**Figure 1:** Mycelium elongation and moisture resistance.

**Figure 2:** The relationship between temperature and mycelial elongation.

**Figure 3:** The relationship between humidity and mycelial elongation.

**Figure 4:** Comparison of different fungi under the same humidity.

**Figure 5:** Changes in humidity of a fungus.

**Figure 6:** Effect of fungus on humidity.

**Figure 7:** Comparison of different fungi at the same temperature.

**Figure 8:** Temperature response of a fungus.

**Figure 9:** Temperature change of another fungus.

**Figure 10:** Fitting image of B-type fungus hypha density with temperature and humidity.

**Figure 11:** Three-dimensional fitting model of type A bacteria.

**Table 1:** Ranking.

Fungus name	Competitive ranking	Mycelial elongation rate	Hypha density
Armillaria	0.281	0.398	0.420
Hyphodontia	0.630	3.590	0.080
Laetiporus	0.342	4.115	0.168
Lentinus	0.569	6.380	0.050
Mycoacia subconspersa	0.569	1.300	0.840
Merulius tremullosus	0.813	10.120	0.050
Phlebiopsis gigantea	0.634	6.105	0.480
Porodisculus pendulus	0.465	4.060	0.320
Phellinus robiniae	0.376	2.220	0.095
Phlebia acerina	0.973	8.510	0.270
Pycnoporus sanguineus	0.697	4.970	0.020
Schizophyllum commune	0.626	3.490	0.560
Tyromyces	0.805	3.880	0.060
Xylobolus subpileatus	0.493	0.770	1.740

**Table 2:** Model fit test.

Variables	Coefficient	Standard deviation	*T*-statistic	Significance
*C*	0.372	0.441	0.843	0.413
*K*	-0.016	0.019	-0.847	0.411
*H*	0.212	0.201	1.056	0.309
Decidability factor			0.087	

**Table 3:** Output results.

SSE	*R*-square	Adjusted *R*-square	RMSE
2.046*e*-34	1	NaN	NaN

**Table 4:** Output results.

SSE	*R*-square	Adjusted *R*-square	RMSE
7.754*e*-33	1	NaN	NaN

**Table 5:** Relevant conditions in five different environments.

Temperature band	*x*_1_	*x*_2_	*x*_3_	*x*_4_	*x*_5_	*x*_6_
Drought	34.5	10%	1848	8	31.4	15%
Semiarid	29.4	25%	5038	12	28.3	28%
Temperate	22.5	55%	10274	24	20.7	51%
Tree coniferous forest	8.6	28%	17893	24	10.2	29%
Tropical rainforest	31.5	68%	23137	48	30.2	65%

**Table 6:** Summary data of type A hyphae and type B hyphae.

Temperature band	*x*_7_	*x*_8_	*x*_9_	*x*_10_
Tree coniferous forest	0.017	0.009	0.023	0.016
Tropical rainforest	0.050	0.030	0.110	0.090
Tree coniferous forest	0.450	0.650	0.430	0.710
Tropical rainforest	0.210	0.270	0.280	0.220
Tree coniferous forest	0.760	0.940	0.740	0.980

**Table 7:** Sample data on the variation of decomposition rate with each factor.

Growth rate	Mycelial density	Humidity resistance	Sulfur, phosphorus content	Temperature	Humidity	Decomposition rate
0.25	0.10	3.46	44.1	18.75	1.955	0.31
0.35	1.02	2.55	36.5	25.85	1.510	0.64
0.21	0.16	4.18	58.6	18.20	2.325	0.47
0.25	0.50	4.64	48.6	18.75	2.491	0.46
0.25	0.65	3.09	13.0	20.40	1.805	0.59
0.49	0.91	4.34	4.7	23.10	2.265	0.51
0.25	0.55	2.85	60.7	25.30	1.670	0.58
0.76	0.61	2.21	44.6	24.75	1.190	0.53
0.77	0.12	1.89	9.1	21.70	1.020	0.47
0.50	0.07	3.65	17.2	24.20	1.935	0.32
1.07	0.63	1.43	8.9	24.20	0.770	0.57
4.71	0.02	1.29	15.7	25.45	0.695	0.23
1.96	0.12	1.28	8.3	18.70	0.685	0.45
4.11	0.09	1.31	6.3	23.15	0.715	0.26
4.70	0.03	1.74	3.8	23.85	1.050	0.24
3.77	0.10	2.28	2.3	23.75	1.355	0.31
5.16	0.04	1.52	46.6	23.55	0.910	0.22
6.38	0.05	1.68	0.3	31.30	0.905	0.21
4.14	0.12	1.63	9.7	26.85	0.895	0.35
3.39	0.41	1.55	21.2	24.45	0.941	0.24
1.30	0.84	1.28	0.1	21.95	0.685	0.41
10.62	0.08	1.31	11.0	25.40	0.715	0.22
9.62	0.02	1.38	2.1	24.90	0.762	0.21
8.04	0.05	1.72	2.0	26.90	0.935	0.32
10.80	0.04	2.81	3.0	24.20	1.544	0.35
4.04	0.03	1.71	3.4	26.00	1.011	0.31
1.54	1.80	1.99	14.4	18.90	1.205	0.67
4.06	0.32	1.58	17.0	24.20	0.960	0.43
2.30	0.07	1.84	14.6	26.85	1.075	0.41
2.14	0.12	1.79	9.4	25.70	1.052	0.46
8.75	0.14	1.29	2.9	22.45	0.695	0.32
8.51	0.27	1.62	0.9	21.10	0.980	0.34
4.97	0.02	2.08	1.4	32.45	1.225	0.25
4.41	0.53	2.67	14.3	27.45	1.570	0.53
2.57	0.59	2.74	16.9	28.70	1.581	0.33
3.88	0.06	1.27	1.8	26.30	0.675	0.32
0.77	1.74	5.25	52.5	19.35	2.770	0.36

## Data Availability

The data used to support the findings of this study are included within the article.
